# Prevalence of Ear, Nose, and Throat Problems in Saudi Arabia: A Cross-Sectional Study

**DOI:** 10.7759/cureus.76927

**Published:** 2025-01-04

**Authors:** Mujtaba A Ali, Wafaa S Taishan, Abdulrahman A Almaymoni, Ibrahim N Al Sulaiman, Turki S Althunayyan, Ziad A Abdullah, Manar Alharbi, Hassan H Alalwani, Thamer M Alzahrani, Gaida Felemban

**Affiliations:** 1 Department of Surgery, Faculty of Medicine, Al Baha University, Al Baha, SAU; 2 Department of Otolaryngology, Faculty of Medicine, Al Baha University, Al Baha, SAU; 3 College of Medicine and Surgrey, King Khalid University, Abha, SAU; 4 College of Medicine, Najran University, Najran, SAU; 5 Department of Medicine and Surgery, Qassim University, Qassim, SAU; 6 Department of Otolaryngology - Head and Neck Surgery, Faculty of Medicine, King Abdulaziz University Hospital, Jeddah, SAU; 7 Department of Radiology, King Faisal Hospital, Makkah, SAU; 8 Department of Otolaryngology, King Fahad Hospital, Al Baha, SAU; 9 Department of Emergency Medicine, King Faisal Hospital, Makkah, SAU

**Keywords:** ent problems, knowledge, prevalence, risk factors, saudi arabia, symptoms

## Abstract

Background

Ear, nose, and throat (ENT) disorders are common and significantly impact the quality of life. This study aimed to assess the prevalence of ENT problems among the Saudi population and to explore its association with sociodemographic factors, knowledge, and healthcare utilization.

Methodology

A cross-sectional study was conducted among 405 participants aged 18-80 years across Saudi Arabia. Data were collected using a self-administered, anonymous electronic questionnaire distributed through social platforms. Data was cleaned on Excel (Microsoft® Corp., Redmond, WA, USA) and analyzed using IBM SPSS Statistics for Windows, Version 27 (Released 2020; IBM Corp., Armonk, NY, USA).

Results

The study revealed that 38.5% of participants were diagnosed with a chronic ENT condition, with sinusitis being the most common (n = 90, or 22.2%). Chronic nasal congestion (n = 187, or 46.2%), tinnitus (n = 182, or 44.9%), and hoarseness (n = 176, or 43.5%) were the most frequently reported symptoms. Significant differences in total ENT problem scores were observed based on gender, with females having higher median scores than males (p = 0.038). Knowledge of ENT problems was rated as average by 213 (52.6%) participants, with 376 (92.8%) supporting the need for public awareness campaigns. Healthcare utilization showed that 164 (40.5%) sought medical care over the past year, while 178 (44.0%) visited an otolaryngologist for ENT symptoms.

Conclusion

The study highlights a high prevalence of ENT problems in Saudi Arabia, particularly among the female population. There is a need for targeted public health interventions and educational campaigns to improve the awareness of the population, and to reduce the burden of ENT disorders. Future research should focus on longitudinal studies to explore causal relationships between risk factors and ENT conditions.

## Introduction

A category of illnesses that impact the ear, nose, and throat (ENT) is known as ENT disorders. In addition, it's called otolaryngology (ORL) [1]. They are very common, often cause major disruptions in the lives of those who experience them, and are often treated in an emergency department (ED) [2]. However, because ENT illnesses might have morbidities that affect physiological function, they are extremely important [3]. The specialty area of medicine known as ORL, or ENT medicine, focuses on the diagnosis and treatment of conditions affecting the head and neck, as well as the ENT. It is impossible to exaggerate how important it is for the general public to be aware of ORLs because many common ENT problems have a substantial influence on a person's quality of life and can cause more serious issues if left untreated [4,5]. These issues include taste, smell, speaking, breathing, swallowing, phonation, lower respiratory tract protection, hearing, and secretion clearance [6,7]. Symptoms related to ENT disorders are among the most common reasons people contact primary care physicians worldwide [8,9]. Concern over younger people's knowledge and awareness of ORL-related concerns is on the rise in Saudi Arabia. This worry stems from the rising number of ENT issues in the nation, where tonsillitis, otitis media, and sinusitis are commonly reported among the populace [10].

Despite the fact that ENT problems are among the most common causes of general practitioner (GP) visits [11,12], the percentage of symptoms that are present varies depending on the symptom and could alter over time if actions or access to medical services vary. To characterize the scope of unreported problems, current prevalence figures are required [13]. Therefore, the purpose of this study was to determine how common ENT complaints are among the population of Saudi Arabia and whether they see a GP, an otolaryngologist, or a hospital for treatment.

## Materials and methods

Study design

A cross-sectional survey was conducted from May 1, 2024, to August 10, 2024, and took place in the Central, Western, Southern, Eastern, and Northern regions of Saudi Arabia. The aim was to estimate the prevalence of ENT problems among the Saudi population and their relation to the area of residency, investigate potential risk factors for ENT problems, and assess the public's knowledge and awareness of ENT problems in Saudi Arabia.

Inclusion and exclusion criteria

We encompassed both male and female, Saudi and non-Saudi individuals living in Saudi Arabia, aged between 18 and 80 years, who agreed to participate in the current survey. Populations who do not live in Saudi Arabia, or who are under 18 or above 80 years of age, and those who did not agree to participate, were excluded.

Sample size

The estimated sample size, according to Cochran's equation, is about 385, with a precision level of ±5% and a confidence level of 95%. The study enlisted 405 participants.

Sampling frame

Data was collected using an anonymous, self-administered, reliable, and validated electronic questionnaire, which was modified to meet the study objectives [14]. The questionnaire was distributed among the general population of Saudi Arabia through social platforms such as WhatsApp and Telegram. All participants were informed in detail about the study aims and data confidentiality. The questionnaire required consent from participants to participate in this study. It has two language versions, English and Arabic, allowing participants to choose the language they feel most comfortable with. The questionnaire is composed of socio-demographic data, information on how common ENT complaints are in Saudi Arabia, risk factors, knowledge and awareness of ENT problems, and ENT (ORL) clinic and specialist utilization.

Statistical analysis plan

This study aimed to estimate the prevalence of ENT problems in Saudi Arabia and to investigate its potential risk factors. The analysis involved both descriptive and inferential statistics. Descriptive statistics were used to summarize and describe the characteristics of the study participants and their responses. Frequencies and percentages were calculated for categorical variables. For continuous variables, medians and interquartile ranges (IQRs) were calculated and tabulated. Participants were surveyed on the presence of 15 specific ENT symptoms, categorized into three groups: Ear Symptoms, Nose and Smell Symptoms, and Throat and Speaking Symptoms. A score of 1 was assigned if the participant reported experiencing the symptom within the past 12 months, whereas a score of 0 was assigned if the participant did not report experiencing the symptom. The individual scores for all 15 symptoms were summed to obtain a Total Symptom Score. The total scores were then analyzed to determine any significant associations between them and potential risk factors. The median awareness scores and IQRs were calculated, and the p-values from the Mann-Whitney U test/Kruskal-Wallis test determined whether there were statistically significant differences in scores among the categorical variables. These non-parametric tests were employed owing to the non-normal distribution of the scores, assessed by the application of the Shapiro-Wilk test (p < 0.05). To find out the association between two categorical variables, such as the participant's perception of their knowledge and awareness and sociodemographic features, the Chi-square test and Fisher's Exact test (where the expected count in cells was less than five) were applied. The significance level for all statistical tests was set at p < 0.05, indicating a 95% confidence interval. Data were cleaned in Excel (Microsoft® Corp., Redmond, WA, USA), and all statistical calculations were performed using IBM SPSS Statistics for Windows, Version 27 (Released 2020; IBM Corp., Armonk, NY, USA).

Ethics statement

The study was conducted after obtaining ethical approval on May 29, 2024, from the Institutional Research Board of Al Baha University, Al Baha, Saudi Arabia (REC/SUR/BU-FM/2024/71). The participants were informed about the study aims and assured of data confidentiality, and consent was obtained from each participant before participating in the study.

The participants were informed about the study aims and assured of data confidentiality. Participation was voluntary, and written informed consent was obtained from all participants before data collection.

## Results

A total of 405 participants (Table 1) were included in the study, with a slight majority of 238 individuals (58.8%) being female, while 167 individuals (41.2%) were male. The majority of participants were younger, with 162 (40%) between 18 and 25 years old, followed by 89 (22%) between 26 and 35 years, 76 (18.8%) between 36 and 45 years, 56 (13.8%) between 46 and 55 years, and 22 (5.4%) being 56 years or older. Most participants were Saudi nationals (n = 380, 93.8%), with only 25 (6.2%) being non-Saudis. Regarding marital status, 208 (51.4%) participants were single, 183 (45.2%) were married, while only two individuals (0.5%) were widowed, and 12 individuals (3.0%) were divorced. In terms of income, 174 (43%) of participants were earning less than 5,000 Saudi Riyals per month. About 116 (28.6%) earned between 5,000 and 10,000 Saudi Riyals, 54 (13.3%) earned between 10,001 and 15,000 Saudi Riyals, and 40 (9.9%) earned between 15,001 and 20,000 Saudi Riyals. Only 21 (5.2%) of participants earned more than 20,000 Saudi Riyals per month. Moreover, the majority of participants held a Bachelor's degree (n = 302, or 74.6%), while 81 (20%) had a high school education or lower. A smaller proportion had completed a Master’s degree (n = 16, or 4.0%) or a Doctorate (n = 6, or 1.5%). Geographically, participants were most commonly from the Central region (n = 168, or 41.5%), followed by the Western region (n = 118, or 29.1%), Southern region (n = 78, or 19.3%), Eastern region (n = 37, or 9.1%), and the Northern region (n = 4, or 1.0%).

**Table 1:** Sociodemographic characteristics of participants in the study (N = 405) N: Frequency; SAR: Saudi Riyal

Variable	Answer	N (%)
Gender	Female	238 (58.8%)
	Male	167 (41.2%)
Age (year)	18-25	162 (40.0%)
	26-35	89 (22.0%)
	36-45	76 (18.8%)
	46-55	56 (13.8%)
	56 and above	22 (5.4%)
Nationality	Non-Saudi	25 (6.2%)
	Saudi	380 (93.8%)
Marital status	Single	208 (51.4%)
	Married	183 (45.2%)
	Widowed	2 (0.5%)
	Divorced	12 (3.0%)
Monthly income (SAR)	Less than 5,000	174 (43.0%)
	5,000-10,000	116 (28.6%)
	10,001-15,000	54 (13.3%)
	15,001-20,000	40 (9.9%)
	More than 20,000	21 (5.2%)
Educational level	Bachelor's degree	302 (74.6%)
	Doctorate	6 (1.5%)
	High school or below	81 (20.0%)
	Master's degree	16 (4.0%)
Region	Central region	168 (41.5%)
	Eastern region	37 (9.1%)
	Northern region	4 (1.0%)
	Southern region	78 (19.3%)
	Western region	118 (29.1%)

Table 2 shows that 156 (38.5%) participants reported being diagnosed with a chronic ENT condition, with the most common conditions being sinusitis (n = 90, or 22.2%), allergic rhinitis (n = 48, or 11.9%), and tonsillitis (n = 44, or 10.9%). Other conditions included nasal polyps (n = 4, or 1.0%), otitis media (n = 39, or 9.6%), tinnitus (n = 44, or 6.7%), and chronic ear infections (n = 11, or 2.7%). Despite this, the majority of participants (n = 249, or 61.5%) had not been diagnosed with a chronic ENT condition. Regarding the frequency of ENT problems, 143 (35.3%) of participants reported that they rarely or never experienced these issues, 121 (29.9%) reported experiencing them once or twice a year, 59 (14.6%) reported three to five times a year, and 82 (20.2%) indicated they had ENT problems more than five times a year.

**Table 2:** Ear, nose, and throat conditions experienced by participants N: Frequency

Question	Answer	N (%)
Have you ever been diagnosed with any chronic ear, nose, and throat conditions?	No	249 (61.5%)
	Yes	156 (38.5%)
If yes, what is the condition?	Sinusitis	90 (22.2%)
	Allergic rhinitis	48 (11.9%)
	Nasal polyps	4 (1.0%)
	Tonsillitis	44 (10.9%)
	Otitis media	39 (9.6%)
	Tinnitus	27 (6.7%)
	Chronic ear infections	11 (2.7%)
How often do you suffer from ear, nose, and throat problems?	Rarely or never	143 (35.3%)
	Once or twice a year	121 (29.9%)
	3 to 5 times a year	59 (14.6%)
	More than 5 times a year	82 (20.2%)

The prevalence of various ENT symptoms experienced by participants in the past year is shown in Figure 1. Tinnitus was the most common ear symptom (n = 182, or 44.9%), followed by dizziness or vertigo (n = 152, or 37.5%), recurring ear pain (n = 115, or 28.4%), recurring ear infections (n = 90, or 22.2%), difficulty hearing (n = 79, or 19.5%), and ear discharge (n = 61, or 15.1%). Nasal symptoms were also highly prevalent among the study participants. Chronic nasal congestion affected 187 (46.2%) of participants, making it the most common nasal issue, whereas 105 (25.9%) of participants reported experiencing a loss of smell, while 100 (24.7%) suffered from facial pain, and 57 (14.1%) from recurrent nosebleeds. Regarding throat-related symptoms, 176 (43.5%) participants experienced hoarseness or changes in their voice, followed by chronic sore throats (n = 155, or 38.3%), difficulty swallowing (dysphagia) (n = 151, or 37.3%), and a decrease in their sense of taste (n = 78, or 19.3%). Additionally, 50 (12.3%) participants reported noticing lumps or swelling in their neck or throat.

**Figure 1:** Ear, nose, and throat symptoms experienced by participants in the past year

Figure 2 illustrates participants' perceptions of the risk factors associated with ENT problems. A majority of participants (n = 279, or 68.9%) indicated allergies as a significant risk factor, followed by air pollution (n = 234, or 57.8%), smoking or exposure to second-hand smoke (n = 227, or 56.0%), and recurrent respiratory infections (n = 226, or 55.8%). However, poor oral hygiene was considered a less significant risk factor, with only 98 (24.2%) participants viewing it as a contributor to ENT problems.

**Figure 2:** Participants perceptions regarding risk factors of ear, nose, and throat problems

Participants' knowledge and awareness of ENT problems, as well as their healthcare utilization (Table 3), showed that a significant portion of participants (n = 213, or 52.6%) rated their knowledge and awareness of common ENT issues as average, while only 21 (5.2%) reported their knowledge as high or very high. Despite this, a strong majority (n = 376, or 92.8%) supports enhancing public awareness about ENT diseases through educational campaigns or sessions, and 272 (67.2%) participants were aware of the availability of ENT clinics in their healthcare system. When it comes to healthcare utilization, 164 (40.5%) participants sought medical care for ENT problems in the past year, and 178 (44.0%) visited an otolaryngologist. The primary reasons for seeing an otolaryngologist were ear diseases (n = 160, or 39.5%) and nose diseases (n = 150, or 37.0%), with throat diseases being less common (n = 95, or 23.5%).

**Table 3:** Participants knowledge of ENT problems and healthcare utilization N: Frequency; ENT: Ear, nose, and throat

Question	Answer	N (%)
How would you rate your overall knowledge and awareness of common ENT problems and their management?	Very low	68 (16.8%)
	Low	103 (25.4%)
	Average	213 (52.6%)
	High	15 (3.7%)
	Very high	6 (1.5%)
Do you propose to improve public awareness about ENT diseases through educational campaigns/sessions?	No	29 (7.2%)
	Yes	376 (92.8%)
Are you aware of the availability of ear, nose, and throat clinics and medical facilities in your local healthcare system?	No	133 (32.8%)
	Yes	272 (67.2%)
Have you sought medical care for any ear, nose, and throat problems in the past 12 months?	No	241 (59.5%)
	Yes	164 (40.5%)
Have you visited an otolaryngologist for any ear, nose, and throat symptoms in the past 12 months?	No	227 (56.0%)
	Yes	178 (44.0%)
What was the reason for that?	Ear diseases	96 (39.5%)
	Nose diseases	90 (37.0%)
	Throat diseases	57 (23.5%)

Table 4 presents a comparison of ENT problem scores among different sociodemographic characteristics. Gender was the only sociodemographic factor with a statistically significant difference in ENT problem scores. Females reported a significantly higher median ENT problem score of 4 (IQR: 2-7), compared to males, who had a median score of 3 (IQR: 1-6). The median ENT problem score varied by age group, with younger individuals (18-25 years) reporting a median score of 3 (IQR: 1-6) and older individuals (56 and above) reporting a higher median score of 6 (IQR: 3-8). Non-Saudi participants had a median score of 5 (IQR: 3-7), compared to 4 (IQR: 1-6) for Saudi participants, but these differences were not statistically significant. Similarly, other factors, such as marital status, monthly income, educational level, and geographical area, showed variations in scores, but none reached statistical significance.

**Table 4:** Comparison of ENT problems among sociodemographic characteristics ^a^ denotes p-value; *A p-value <0.05 is considered as statistically significant N: Frequency; SAR: Saudi Riyal; ENT: Ear, nose, and throat; IQR: Interquartile range

Variable	Answer	ENT problems score	Sig.^a^
		Median (IQR)	
Gender	Female	4 (2-7)	0.038*
	Male	3 (1-6)	
Age (year)	18-25	3 (1-6)	0.083
	26-35	4 (2-6)	
	36-45	4 (1-7)	
	46-55	4 (1-7)	
	56 and above	6 (3-8)	
Nationality	Non-Saudi	5 (3-7)	0.066
	Saudi	4 (1-6)	
Marital status	Single	3 (1-6)	0.073
	Married	4 (2-7)	
	Widowed	5 (5-5)	
	Divorced	7 (4-7)	
Monthly income (SAR)	Less than 5,000	4 (1-6)	0.275
	5,000-10,000	4 (2-7)	
	10,001-15,000	4 (2-6)	
	15,001-20,000	3 (2-6)	
	More than 20,000	4 (0-6)	
Educational level	Bachelor's degree	4 (1-6)	0.220
	Doctorate	4 (1-6)	
	High school or below	5 (2-7)	
	Master's degree	3 (1-5)	
Geographical area	Central region	3 (1-6)	0.275
	Eastern region	3 (2-6)	
	Northern region	5 (1-9)	
	Southern region	4 (2-7)	
	Western region	5 (2-7)	

Table 5 compares knowledge and awareness of common ENT problems among different sociodemographic characteristics. Significant differences were found in knowledge levels across gender, nationality, and marital status. Females reported higher levels of high or very high knowledge (n = 24, or 5.9%), compared to males (n = 17, or 4.2%), and a lower level of low or very low knowledge (n = 143, or 35.3% vs. n = 211, or 52.1% for males), with the difference being statistically significant. Non-Saudi participants had higher levels of high knowledge (n = 65, or 16.0%), compared to Saudis (n = 18, or 4.5%). Marital status also showed significant differences, with a slightly higher percentage of married individuals having high or very high knowledge (n = 27, or 6.6% vs. n = 17, or 4.3%), compared to singles. Similarly, singles had a higher percentage of very low or low knowledge (n = 202, or 50.0% vs. n = 137, or 33.9%). Other sociodemographic factors, including age, monthly income, educational level, and geographical area, did not show statistically significant differences in the distribution of knowledge and awareness levels. 

**Table 5:** Comparison of knowledge and awareness among sociodemographic characteristics ^a^ denotes p-value; *A p-value <0.05 is considered as statistically significant N: Frequency; SAR: Saudi Riyal; ENT: Ear, nose, and throat

Variable	Answer	How would you rate your overall knowledge and awareness of common ENT problems and their management?			Sig.^a^
		High or very high	Average	Low or very low	
		N (%)	N (%)	N (%)	
Gender	Female	14 (5.9%)	140 (58.8%)	84 (35.3%)	0.003*
	Male	7 (4.2%)	73 (43.7%)	87 (52.1%)	
Age (year)	18-25	5 (3.1%)	82 (50.6%)	75 (46.3%)	0.313
	26-35	4 (4.5%)	45 (50.6%)	40 (44.9%)	
	36-45	5 (6.6%)	40 (52.6%)	31 (40.8%)	
	46-55	4 (7.1%)	33 (58.9%)	19 (33.9%)	
	56 and above	3 (13.6%)	13 (59.1%)	6 (27.3%)	
Nationality	Non-Saudi	4 (16.0%)	7 (28.0%)	14 (56.0%)	0.006*
	Saudi	17 (4.5%)	206 (54.2%)	157 (41.3%)	
Marital status	Single	9 (4.3%)	95 (45.7%)	104 (50.0%)	0.040*
	Married	12 (6.6%)	109 (59.6%)	62 (33.9%)	
	Widowed	0 (0.0%)	1 (50.0%)	1 (50.0%)	
	Divorced	0 (0.0%)	8 (66.7%)	4 (33.3%)	
Monthly income (SAR)	10,001-15,000	3 (5.6%)	28 (51.9%)	23 (42.6%)	0.443
	15,001-20,000	3 (7.5%)	20 (50.0%)	17 (42.5%)	
	5,000-10,000	2 (1.7%)	62 (53.4%)	52 (44.8%)	
	Less than 5,000	10 (5.7%)	92 (52.9%)	72 (41.4%)	
	More than 20,000	3 (14.3%)	11 (52.4%)	7 (33.3%)	
Educational level	Bachelor's degree	14 (4.6%)	155 (51.3%)	133 (44.0%)	0.254
	Doctorate	1 (16.7%)	4 (66.7%)	1 (16.7%)	
	High school or below	6 (7.4%)	42 (51.9%)	33 (40.7%)	
	Master's degree	0 (0.0%)	12 (75.0%)	4 (25.0%)	
Geographical area	Central region	7 (4.2%)	85 (50.6%)	76 (45.2%)	0.742
	Eastern region	3 (8.1%)	22 (59.5%)	12 (32.4%)	
	Northern region	0 (0.0%)	1 (25.0%)	3 (75.0%)	
	Southern region	5 (6.4%)	42 (53.8%)	31 (39.7%)	
	Western region	6 (5.1%)	63 (53.4%)	49 (41.5%)	

## Discussion

The main aim of this cross-sectional study was to assess the prevalence of ENT problems among the population in Saudi Arabia. In our study, the sociodemographic characteristics of the participants provide context for understanding the prevalence of ENT conditions. The majority of participants were female (58.8%), younger in age, and primarily from the Central and Western regions of Saudi Arabia. This demographic profile is significant because previous studies have suggested that women and younger adults are more likely to report ENT symptoms, possibly due to higher health awareness and care-seeking behaviors [15]. Furthermore, the relationship between income and ENT health, suggested by the higher frequency of ENT problems among participants with lower income, aligns with existing literature that links economic status with health outcomes, due to factors like access to healthcare and environmental exposures [16].

Our study's results show that a significant proportion of the participants (5%) had been diagnosed with a chronic ENT condition, with sinusitis (22.2%) being the most common diagnosis, which is higher than the percentage reported by Fokkens et al. (2012) among European populations (10%-15%) [17]. These findings align with previous research conducted in the Middle East, where sinusitis is reported as a prevalent condition, particularly in regions with high exposure to environmental pollutants and allergens. For instance, a study by Homood et al. (2017) reported a similarly high prevalence of sinusitis in Saudi Arabia, emphasizing the role of environmental factors in its occurrence [18]. The prevalence of allergic rhinitis, at 11.9%, in our study closely matches the 12% reported in Middle Eastern populations, suggesting a consistent burden of this condition across similar climatic regions [19]. Regarding the frequency of ENT problems, our study revealed that 20.2% of participants reported complaints more than five times a year, a figure that is higher than that found in other international studies. A study conducted by Leland et al. (2021) found that chronic ENT conditions, like rhinitis and sinusitis, typically exacerbate more frequently under environmental stressors prevalent in urban areas - a finding that might explain the higher incidence in our pool from the Central and Western regions of Saudi Arabia [20].

The data in Figure 1 highlight the prevalence of various ENT symptoms experienced by participants over the past year. Tinnitus, experienced by 44.9% of participants, emerged as the most common ear-related symptom. This finding is consistent with other studies in the region and globally, which report tinnitus as a prevalent condition, often associated with noise exposure, age-related hearing loss, and other underlying health issues. For instance, a study by Henry et al. (2020) [21] found that tinnitus affects approximately 10%-15% of the adult population worldwide, with higher prevalence rates observed in regions with significant noise pollution or occupational hazards. Chronic nasal congestion, reported by 46.2% of our subjects, similarly exceeds figures observed in other studies, where prevalence rates generally hover around 20%-30% [22]. This may potentially be linked to environmental factors, such as air quality, which is known to impact nasal congestion rates, particularly in urban areas [23]. The rate of hoarseness, at 43.5%, is significantly higher than the estimates reported by Alrahim et al. (2018), who found that about 5%-10% of the population experiences voice disorders annually [24]. Dysphagia, affecting 37.3% of participants, is substantially higher than the prevalence usually reported in the literature, where it affects approximately 7% of the general population, mostly older adults [25]. Moreover, the study found that 37.5% of participants experienced dizziness or vertigo, which is consistent with findings from other studies that have reported vertigo as a common symptom, particularly in older adults or those with underlying vestibular disorders. For example, a study identified vertigo as a frequent complaint in primary care settings, often associated with vestibular migraines, benign paroxysmal positional vertigo (BPPV), and other inner ear conditions [26]. Finally, the relatively lower prevalence of symptoms like ear discharge (15.1%) and lumps or swelling in the neck or throat (12.3%) is consistent with the fact that these symptoms are typically associated with more severe or advanced ENT conditions, such as infections or malignancies, which are less common in the general population. This observation aligns with the findings by Chiong et al. (2020), who noted that while these symptoms are concerning, they tend to occur less frequently in the absence of serious disease [27].

The data in Figure 2 indicate that most participants identified allergies (68.9%) as the primary risk factor for ENT problems, followed by air pollution (57.8%), smoking or second-hand smoke exposure (56.0%), and recurrent respiratory infections (55.8%). These perceptions align with existing studies that link these factors to the prevalence of ENT conditions like allergic rhinitis, sinusitis, and chronic bronchitis [28,29]. Interestingly, only 24.2% recognized poor oral hygiene as a significant risk, despite research suggesting its role in ENT health [10]. This discrepancy highlights an area where public awareness could be improved.

Our findings suggest a moderate level of knowledge and awareness of ENT problems among the study participants, with a significant majority (52.6%) rating their knowledge as average, and only a small fraction (5.2%) considering their awareness to be high or very high. This finding aligns with studies that reported similar trends of moderate awareness of ENT issues among general populations in other regions [3,30]. The study highlights a potential gap in understanding ENT health, which is critical for early diagnosis and treatment. Despite this, there is strong support (92.8%) for improving public awareness through educational campaigns, reflecting a positive attitude towards enhancing knowledge in this area. Awareness of available ENT clinics was relatively high (67.2%), which is encouraging, but the fact that 32.8% of participants were unaware of these services points to an ongoing need for better dissemination of healthcare information.

Regarding healthcare utilization, 40.5% of the participants sought medical care for ENT problems within the past year, and 44.0% visited an otolaryngologist - figures that are slightly higher than the rates observed in other regional studies, such as the one by Batool et al. (2023), which reported approximately 30% of participants seeking specialist ENT consultations [31]. The higher consultation rates in our study could be attributed to better healthcare access or possibly higher health awareness among our participants. The present study shows that women had significantly higher ENT problem scores compared to males (median score of 4 for females and 3 for males), which is consistent with other studies that suggest women are more likely to report ENT symptoms and seek medical attention for these issues [16]. The variation in ENT problem scores by age also aligns with existing research, with older participants (56 and above) reporting higher scores, reflecting the increased prevalence of ENT issues with age [23]. While differences in ENT problem scores by nationality, marital status, income, education, and geographical area were observed, none of these factors reached statistical significance. This suggests that, while sociodemographic factors may influence the prevalence of ENT problems, they are not the sole determinants, and other factors, such as environmental exposures and access to healthcare, likely play a crucial role [32].

The findings of the present study show that females had higher levels of knowledge and awareness compared to males. This aligns with existing literature, where women often demonstrate greater health literacy and are more proactive in seeking health-related information than men [15]. The data also show that non-Saudi participants had a higher percentage of high knowledge (16.0%) compared to Saudi counterparts (4.5%), a significant difference that might be influenced by the diverse educational backgrounds and access to health information among expatriates versus locals. This finding contrasts with some studies, which found that locals often have better access to healthcare resources. However, it is possible that non-Saudis in this study are more proactive in acquiring health knowledge due to being in a foreign country, emphasizing the importance of context in health literacy [23]. Marital status also played a role, with married individuals showing slightly higher levels of high or very high knowledge (6.6%) compared to single ones (4.3%). This trend is consistent with studies suggesting that married individuals may have better health knowledge and behaviors, possibly due to mutual support and shared health responsibilities within marriage [14]. Other sociodemographic factors, such as age, income, educational level, and geographical area, did not show statistically significant differences in knowledge and awareness.

Limitations of the study

This study has several limitations that should be considered when interpreting the results. Firstly, the use of a self-administered electronic questionnaire may have introduced response bias, as participants might have over- or under-reported their symptoms and knowledge levels. Additionally, the study's cross-sectional design only captures a snapshot in time, limiting our ability to establish causal relationships between risk factors and ENT problems. The sample, while representative of the general population, may not fully account for regional variations in healthcare access and environmental exposures across different areas of Saudi Arabia. Furthermore, the reliance on self-reported data for medical diagnoses and healthcare utilization could have led to inaccuracies, as these reports were not independently verified by medical records.

## Conclusions

The significant prevalence of ENT problems among the Saudi Arabian population, particularly in relation to sociodemographic factors, underlines the need for improved public awareness and healthcare access. Common conditions like sinusitis, allergic rhinitis, and tinnitus were prevalent, highlighting areas where targeted interventions could make a difference. To build on these findings, future research should explore longitudinal studies to better understand the causal relationships between risk factors and ENT conditions. Moreover, public health initiatives and educational campaigns focused on specific demographics, such as men and lower-income groups, could play a crucial role in reducing the burden of ENT problems and enhancing overall public health in Saudi Arabia.

## Appendices

**Table 6:** Research questionnaire

Answer	Demographic information
Male	Gender
Female	
18-25	Age (year)
26-35	
36-45	
46-55	
56 and above	
Single	Marital status
Married	
Divorced	
Widowed	
Saudi	Nationality
Non-Saudi	
High school or below	Educational level
Bachelor's degree	
Master's degree	
Doctorate degree	
Less than 5,000	Monthly income (SAR)
5,000-10,000	
10,001-15,000	
15,001-20,000	
Above 20,000	
Central region	From which region are you from
Eastern region	
Western region	
Southern region	
Northern region	
Answer	ENT-related symptoms question
Yes	Have you ever been diagnosed with a chronic ENT condition?
No	
Sinus infections	If yes, which of the following ENT conditions have you been diagnosed with? (Select all that apply)
Sinusitis	
Nasal polyps	
Allergic rhinitis	
Tonsillitis	
Hearing tinnitus	
Otitis media	
Chronic ear infections	
Others….specify	
Rarely or never	How often do you experience any ENT (Ear, Nose, and Throat) related problems?
1-2 times per year	
3-5 times per year	
More than 5 times per year	
Yes	Have you ever experienced any Ear discharge in the past year?
No	
Yes	Have you had any recurrent ear infections in the past year?
No	
Yes	Have you had any recurrent ear pain in the past year?
No	
Yes	Have you noticed any ringing or buzzing sounds in your ears (tinnitus) in the past year?
No	
Yes	Have you experienced any difficulty hearing in the past year?
No	
Yes	Have you experienced any spinning around (vertigo) in the past year?
No	
Yes	Have you experienced persistent nasal congestion (stuffiness) in the past year?
No	
Yes	Have you had any facial pain in the past year?
No	
Yes	Have you had any recurrent nosebleeds (epistaxis) in the past year?
No	
Yes	Have you noticed any changes in your sense of smell (anosmia) in the past year?
No	
Yes	Have you had any decrease with your sense of taste in the past year?
No	
Yes	Have you experienced any persistent sore throat in the past year?
No	
Yes	Have you experienced any voice changes, (hoarseness) in the past year?
No	
Yes	Have you had any difficulty swallowing (dysphagia) in the past year?
No	
Yes	Have you noticed any lumps, swelling, or masses in your neck or throat in the past year?
No	
Answer	Risk factors for ENT problems
Air pollution	Which of the following factors do you believe may contribute to ENT problems? (Select all that apply)
Smoking or secondhand smoke exposure	
Allergies	
Frequent respiratory infections	
Poor oral hygiene	
Answer	Knowledge and awareness of ENT problems: How would you rate your overall knowledge and awareness of common ENT problems and their management?
Very low	
Low	
Moderate	
High	
Very high	
Answer	ENT (Otolaryngology) Clinic and Specialist Utilization
Yes	Are you aware of the availability of specialized ENT (Otolaryngology) clinics and services in your local healthcare system?
No	
Yes	Have you sought medical attention for any ENT-related issues in the past 12 months?
No	
Yes	Have you visited an Otolaryngologist for any ENT symptoms in the past 12 months?
No	
Ear disease	What was the reason for that?
Nose disease	
Throat disease	
